# Pore Strategy Design of a Novel NiTi-Nb Biomedical Porous Scaffold Based on a Triply Periodic Minimal Surface

**DOI:** 10.3389/fbioe.2022.910475

**Published:** 2022-06-08

**Authors:** Yuting Lv, Guohao Liu, Binghao Wang, Yujin Tang, Zhengjie Lin, Jia Liu, Guijiang Wei, Liqiang Wang

**Affiliations:** ^1^ College of Mechanical and Electronic Engineering, Shandong University of Science and Technology, Qingdao, China; ^2^ State Key Laboratory of Metal Matrix Composites, Shanghai Jiao Tong University, Shanghai, China; ^3^ Affiliated Hospital of Youjiang Medical University for Nationalities, Baise, China; ^4^ 3D Printing Clinical Translational and Regenerative Medicine Center, Shenzhen Shekou People’s Hospital, Shenzhen, China

**Keywords:** additive manufacturing, triply periodic minimal surfaces, NiTi-Nb, porous scaffolds, pore strategy

## Abstract

The pore strategy is one of the important factors affecting the biomedical porous scaffold at the same porosity. In this work, porous scaffolds were designed based on the triply periodic minimal surface (TPMS) structure under the same porosity and different pore strategies (pore size and size continuous gradient distribution) and were successfully prepared using a novel Ni_46.5_Ti_44.5_Nb_9_ alloy and selective laser melting (SLM) technology. After that, the effects of the pore strategies on the microstructure, mechanical properties, and permeability of porous scaffolds were systematically investigated. The results showed that the Ni_46.5_Ti_44.5_Nb_9_ scaffolds have a low elastic modulus (0.80–1.05 GPa) and a high ductility (15.3–19.1%) compared with previous works. The pore size has little effect on their mechanical properties, but increasing the pore size significantly improves the permeability due to the decrease in specific surfaces. The continuous gradient distribution of the pore size changes the material distribution of the scaffold, and the smaller porosity structure has a better load-bearing capacity and contributes primarily to the high compression strength. The local high porosity structure bears more fluid flow, which can improve the permeability of the overall scaffold. This work can provide theoretical guidance for the design of porous scaffolds.

## Introduction

Biomedical metal materials are one of the ideal materials for treating bone defects because of their high strength, corrosion resistance, and biocompatibility (Wang et al., 2020; Guo et al., 2022), but the solid metal material has a much higher elastic modulus than that of human bone, easily resulting in “stress shielding” and degradation of the bone tissue around the implant (Geetha et al., 2009). The porous scaffolds can be used to replace the solid materials, which can not only reduce the elastic modulus but can also promote cell adhesion and the growth of bone tissue (Chen et al., 2020; Mao et al., 2022). The traditional processing methods are difficult to achieve the preparation of complex porous structures, limiting the development of metal porous scaffolds. The development of additive manufacturing technology provides a solution for the preparation of complex porous structures. Additive manufacturing can both personalize bone scaffolds with precise dimensions to match the shape of the bone defect and precisely control their porosity, pore size, and distribution (Wang et al., 2020). Therefore, additive manufacturing of metal porous scaffolds has great potential in the field of bone defect treatment.

The structure design of porous scaffolds is one of the focuses of scientists in various countries. Previous studies have mainly focused on lattice structures based on the CAD method and topology optimization (Wang et al., 2016; Wang et al., 2019). The common types of lattice structural units are the diamond structure (Zhang et al., 2018; Cutolo et al., 2020; Li et al., 2020), body-centered cubic (BCC) structure (Arabnejad et al., 2016; Li et al., 2019), and dodecahedral structure (Liu et al., 2017; Guo et al., 2020). However, the lattice structures have an uneven transition of structural units, stress concentration, and difficult parametric design, which makes it difficult to meet the requirements of high-performance porous scaffolds (Giannitelli et al., 2014). Triply periodic minimal surfaces (TPMSs) are surfaces with the periodic distribution of zero mean curvature in three-dimensional space (Yuan et al., 2019). Zhang et al. (2020)designed a Ti6Al4V scaffold with a single directional gradient variation by changing the minimal surface equation and found that the scaffold had good mechanical properties and permeability matching those of natural bone tissue. Previous investigations have indicated that the minimal surface method has significant advantages in improving the mechanical properties and parametric design of scaffolds (Lv et al., 2021).

The human bone has a porous structure, and the different areas have various pore sizes and size distribution (Onal et al., 2018). The porous scaffold prepared by different pore strategies can be used to simulate human bone pore size features. Ran et al. (2018) found that the mechanical properties of the scaffolds decreased with the increase in the pore size and porosity, and the small pore was favorable for cell adhesion, and the large pore was favorable for cell proliferation; when the pore size was 600 μm, the scaffolds showed the optimal bone tissue growing-in ability. Therefore, from the present investigations, increasing the pore size or porosity can match the biomechanical properties of bone tissue and improve the biological properties of the scaffold (Ouyang et al., 2019). Under the same porosity, the pore strategy is the main factor affecting the mechanical properties and permeability of porous scaffolds, which includes pore size and pore size distribution. However, as far as we know, the effect of pore strategy based on the triply periodic minimal surface structure on the mechanical properties and permeability of porous scaffolds has rarely been mentioned.

NiTi system alloy has superelasticity, shape-memory function, good biocompatibility, and corrosion resistance; thus it is a good functional biomedical material (Habijan et al., 2012; Li et al., 2014). However, the Ni_4_Ti_3_ second phase in the NiTi alloy reduces the toughness and ductility of the alloy, so it is necessary to introduce a high strength second phase to improve the mechanical properties. It is well-known that Nb is a typical wide hysteresis phase transformation element and also has good biocompatibility. Therefore, the addition of Nb can not only change the microstructures (Lin et al., 2013; Gu et al., 2019) but can also improve the biocompatibility of NiTi alloy (Guo et al., 2021). The research on the additive manufactured NiTi-Nb alloy is still in the initial stage, and it is mainly prepared as a bulk alloy. Liu et al. (2020) prepared NiTi-Nb eutectic bulk alloy by additive manufacturing and found that Nb particles could accelerate the eutectic phase transition and the precipitation of the β-Nb phase, which improved the mechanical properties of the scaffold. However, the study of additive manufacturing of NiTi-Nb porous scaffolds has not been reported.

Therefore, in this work, the porous scaffolds were designed and simulated by human bone pore size features based on minimal surface structures under the same porosity and different pore strategies, including uniform scaffolds with different pore sizes and scaffolds with continuous gradient distribution of pore sizes. The porous scaffolds were successfully prepared using a novel Ni_46.5_Ti_44.5_Nb_9_ alloy and selective laser melting (SLM) technology, and the effects of the pore strategies on the formability, mechanical properties, and permeability of the porous scaffolds were systematically investigated.

## Materials and Methods

### Design and Preparation of the Scaffolds

In this work, porous scaffolds with the same porosity and different pore strategies were obtained by controlling minimal surface structural units, including three uniform distributed porous scaffolds with different pore sizes (500, 750, and 900 μm) and two porous scaffolds with a gradient distribution of pore sizes along the radial direction (pore sizes of 500–900 μm from inside to outside and 900–500 μm from inside to outside). Correspondingly, the scaffolds were named G500, G750, G900, G500-900, and G900-500, and the designed models are shown in Figure 1.

**FIGURE 1:** Design model of the scaffold.

The G-structure of the minimal surface was selected to prepare the scaffolds. The equation of the G-structure is as follows:

$$\varphi {\left(x,y,z\right)}_{G}=\sin\left(\frac{2\pi }{L}x\right)\cos\left(\frac{2\pi }{L}y\right)+\sin\left(\frac{2\pi }{L}z\right)\cos\left(\frac{2\pi }{L}x\right)+\sin\left(\frac{2\pi }{L}y\right)\cos\left(\frac{2\pi }{L}z\right)=\mathrm{C,}$$

where L is the period of the minimal surface, i.e., the structure unit size, and C is the threshold, which is used to control the volume of the solid part. At a certain L, the pore size varies over the range (0, L). The structural unit sizes of the uniform scaffolds are 0.845, 1.242, and 1.522 mm, respectively (Figure 1). Furthermore, when the C value is replaced with a function related to the radius, a pore size distribution with continuous gradient variation in the radial direction can be obtained. The internal and external porosities (C_in,_ C_out_) of the G500-900 scaffold are 41 and 90%, respectively, and the opposite is true for the G900-500 scaffold. Eventually, the porosity distribution function of the G-structure is as follows:

$$C_{\left(\mathrm{x,y}\right)}=\left(C_{\mathrm{out}}-C_{\mathrm{in}}\right){\left(\frac{\sqrt{x^{2}+y^{2}}}{r}\right)}^{n}+C_{\mathrm{in}},$$

The G-structure equations and pore size distribution functions were imported into Mathematica soft to generate the model with a height of 15 mm and a diameter of 10 mm, and then, the models were repaired by importing into MagicSoft before SLM preparation.

NiTi alloy powder and Nb powder were used as raw materials, and the powder ratio was 91:9. Thus, the nominal chemical composition of the blended powder was Ni_46.5_Ti_44.5_Nb_9_. After a high-energy ball mill for 3 h, the blended powder was used to prepare the scaffolds by SLM. The processing parameters were set as follows: the laser power was 200 W, powder layer thickness was 30 μm, spot size was 120 μm, laser scanning speed was 600 mm/s, scanning direction rotated 67° between successive layers, and substrate preheating temperature was 160°C. The scaffolds were washed three times with anhydrous ethanol in an ultrasonic cleaner to remove the unmelted metal powder from the surface.

### Macro Morphologies and Microstructure Observation

The Archimedes method and dry weight method were used to calculate the density and porosity of the scaffolds. Micro-CT (PerkinElmer, Quantum GX II) was used to observe the macroscopic morphology of the scaffolds. The scanning voltage and current were 90 Kv and 80 μA, respectively, and the scanning time was 14 min. The 3D reconstruction was carried out using the device’s built-in software with the same threshold values. A scanning electron microscope (SEM, JSM-7600F, JEOL) was used to observe the surface morphology and microstructure of the scaffolds. For the microstructure observation, the samples were ground and polished to a mirror finish by standard metallographic procedures and etched by using a reagent (composed of 10 vol% HNO_3_, 20 vol% HF, and 70 vol% H_2_O) for 15 s.

### Compression Tests and Finite Element Simulation

Compression tests were carried out by using an MTS servo-hydraulic press (MTS 810, MTS, USA) at room temperature and a rate of 0.5 mm/min. The elastic modulus, compression strength, and maximum strain of the scaffolds were calculated based on the stress–strain curves.

The mechanical analysis of the G-structure unit with different porosities and the porous scaffolds was performed by ANSYS 16.0. The mesh type for the finite element analysis was a tetrahedral mesh with a size of 0.1 mm. The material model is chosen to be a nonlinear material, which needs to be created in ANSYS software. The material had an elastic modulus of 37 GPa, a compressive strength of 960 MPa, a Poisson’s ratio of 0.3, a density of 6,475 kg/m^3^, a bulk modulus of 36 GPa, and a shear modulus of 14 GPa. The boundary conditions were set as follows: fixing the bottom of the scaffold, applying a 10% displacement load on the top of the scaffold, and a compression rate of 0.5 mm/min. After the finite element analysis, the stress distribution of the scaffold was the output.

### Permeability Tests and Fluid Finite Element Simulation

In order to evaluate the permeability of the scaffold, the permeability was tested by the falling head method, and the schematic diagram of the device is shown in Figure 2A. In the course of the experiment, the water level in the seepage tube gradually drops from h_1_ to h_2_, which was kept constant for each test. The permeability K of the scaffolds was calculated from the equation of Darcy’s law:

$$K=\frac{\mu HA}{\rho gta}\ln\left(\frac{h_{1}}{h_{2}}\right),$$

where H is the height of the scaffold, A is the cross-sectional areas of the seepage tube, a is the cross-sectional areas of the scaffold, μ is the viscosity of the water, ρ is the density of the water, and g is the acceleration of gravity.

**FIGURE 2:** Permeability experiments and finite element simulations: **(A)** schematic representation of the experimental device used in the falling head permeability test, **(B)** scaffold model, **(C)** model for finite element simulation, and **(D)** boundary setting for finite element simulation.

In order to simulate the flow of human body fluids inside the porous scaffold, ANSYS software was used to simulate the permeability of the scaffold using human body fluid as media, as shown in Figures 2B–D. The density of the fluid was 1,050 Kg/m^3^, the viscosity was 0.0035 Pa٠s, the inlet flow velocity was set to 0.01 m/s, and the outlet pressure was set to 0 Pa (Truscello et al., 2012). After the finite element simulation, the inlet pressure was calculated, and the pressure distribution cloud and flow velocity distribution of the fluid model were the output.

## Results and Discussion

### Macroscopic Morphology Analysis

Figure 3A shows the macroscopic morphologies of the Ni_46.5_Ti_44.5_Nb_9_ porous scaffolds. As can be seen, except for the G900-500 scaffold, all the scaffolds are structurally intact with no obvious defects. The height and the diameter of the scaffolds are 15.11 ± 0.12 mm and 10.06 ± 0.08 mm, respectively, which are basically consistent with the designed model. The density of the porous scaffold measured by the Archimedes drainage method is 6.62 g/cm^3^. The porosity of the scaffold was calculated by the dry weight method and Micro-CT built-in software, as shown in Table 1. The porosity of the porous scaffold is basically consistent with the designed porosity. The surface area of the scaffold model is also obtained by Magics software (Table 1), and it can be found that the surface area of the scaffold increases with the decrease in the pore size. Figure 3B shows the Micro-CT 3D reconstruction image of the porous scaffold, and the results indicated that the prepared porous scaffold has good connectivity, and no pore blockage occurs.

**FIGURE 3:** **(A)** Macroscopic morphologies of Ni_46.5_Ti_44.5_Nb_9_ porous scaffolds and **(B)** micro-CT 3D reconstruction model of the scaffolds.

**TABLE 1:** Modeling parameters and actual porosity of the scaffolds.

Scaffold	Superficial area (mm^2^)	Design mean porosity (%)	Dry weighing porosity (%)	Porosity of the micro-CT reconstruction model (%)
G500	4169.366	70	71.83 ± 0.41	70.28 ± 0.74
G750	2866.860	70	71.07 ± 0.39	67.92 ± 0.21
G900	2367.944	70	68.97 ± 0.31	70.85 ± 0.29
G500-900	2644.182	70	71.67 ± 0.54	67.42 ± 0.53
G900-500	2837.003	70	71.68 ± 0.66	69.01 ± 0.33

Figures 4A–C show SEM images of the surface morphology of the porous scaffolds with pore size strategy. As can be seen, the surface of the Ni_46.5_Ti_44.5_Nb_9_ porous scaffold is uneven and has an obvious step effect (Cheng et al., 2014). The support thicknesses of the scaffolds are found to be larger than the designed dimensions, and the dimensional errors are between 5 and 25%. It should be noted that the center of the G900-500 scaffold shows defect, and the support thickness is also much smaller than the design size (200 μm) (Figure 4D), which is due to the fact that the minimum support thickness of the G900-500 scaffold (200 μm) is close to the processing limit of the SLM (80–250 μm) (Tofail et al., 2018), which lead to the generation of cracks. Therefore, the accuracy of the processing and the minimum design size of the scaffold should be considered in the design of the scaffold. Figures 4E,F show the surface morphology of the G500-900 scaffold, it can be found that the gradient structure of the scaffold varies significantly.

**FIGURE 4:** Surface morphologies of the scaffolds: **(A)** G500, **(B)** G750, **(C)** G900, **(D)** G900-500, **(E)** and **(F)** G500-900.

### Compression Property Analysis

Figure 5 illustrates the macroscopic shape and compression performance of Ni_46.5_Ti_44.5_Nb_9_ scaffolds after compression tests. As can be seen from Figure 5A, the angle between the fracture surface and the loading direction is 45°; this is because the scaffolds are subjected to shear stress during the compression process (Yan et al., 2015; Liu et al., 2018). The compressive stress–strain curves of the Ni_46.5_Ti_44.5_Nb_9_ scaffolds are shown in Figure 5B. Due to the small thickness of support in the G500 scaffold (280 μm), when the stress reached the compressive strength of the scaffold, the local support broke first during the compression process, and the stress dropped sharply. However, the scaffold was not completely broken but was gradually compacted (as shown in Figure 5A), and the stress increased again, resulting in stress fluctuation of compressive curves. The mechanical properties of the Ni_46.5_Ti_44.5_Nb_9_ porous scaffold are listed in Table 2 from which it can be seen that the scaffold has an elastic modulus between 0.80–1.05 GPa, a compressive strength between 42.3–65.8 MPa, and an elongation between 15.3–19.1%. With the same porosity, the difference in mechanical properties of uniform scaffolds with different pore sizes is not significant, indicating that the pore size strategy has little effect on mechanical properties. However, the compression strength of G500-900 and G900-500 scaffolds is significantly higher than that of uniform scaffolds. This is because the radial gradient strategy increases the local support thickness of the scaffolds and improves their load-bearing capacity.

**FIGURE 5:** Compression properties of the scaffolds: **(A)** morphologies of the post-compression test, **(B)** compression stress–strain curve, and **(C)** comparison of mechanical properties of the scaffold with different materials under similar porosity (Sevilla et al., 2007; Ataee et al., 2018; Cutolo et al., 2018; Cutolo et al., 2020; Liu et al., 2020; Luo et al., 2020).

**TABLE 2:** Mechanical properties of Ni_46.5_Ti_44.5_Nb_9_ scaffolds.

Scaffold	Elastic modulus (GPa)	Compression strength (MPa)	Maximum strain (%)
G500	0.86 ± 0.11	42.3 ± 0.9	17.5 ± 0.3
G750	1.03 ± 0.09	49.3 ± 0.6	18.2 ± 0.5
G900	0.80 ± 0.10	47.7 ± 0.9	18.4 ± 0.5
G500-900	0.96 ± 0.06	65.8 ± 1.6	19.1 ± 0.8
G900-500	1.05 ± 0.05	64.4 ± 0.8	15.3 ± 0.7

Figure 5C shows the mechanical properties of porous scaffolds of different materials with similar porosity. As can be seen, the Ni_46.5_Ti_44.5_Nb_9_ scaffolds have higher compressive strength than most of the scaffolds of other materials and also have a high elongation (comparable to CoCr and Ti scaffolds). The Ni_46.5_Ti_44.5_Nb_9_ porous scaffold with 70% porosity has an elastic modulus matching cancellous bone (0.02–2 GPa) and higher compressive strength than cancellous bone, meeting the performance requirements of bone implants (Sevilla et al., 2007). Lu et al. (2021) also prepared porous scaffolds by SLM using the NiTi shape memory alloy. The elastic modulus of the scaffolds with a porosity of 66% was 1.75–2.45 GPa, which could match cancellous bone and avoid stress masking. The NiTi porous scaffold also has good elongation and superelasticity with a maximum recoverable strain of 5.1%. Therefore, NiTi-based porous scaffolds with high porosity have good potential for cancellous bone repairing.

The elastic modulus of the G-structure unit with different porosities was calculated by the finite element simulation software, and the results are shown in Table 3. It can be found that the elastic modulus of the G-structure unit gradually decreases with the increase in porosity, which is consistent with the results obtained by Bartolomeu et al. (2020). The porous scaffolds with different pore size distribution strategies have different porosities. The mechanical properties of the G500-900 scaffold gradually decrease as the porosity increases from the center of the scaffold to the outside. As the porosity of the G900-500 scaffold gradually decreases from the center to the outside of the scaffold, the mechanical properties of gradient scaffolds change gradually along the radius direction. Figure 6 shows the stress distribution in the scaffolds after the compression simulation. We can also observe that the stress in the uniform scaffolds is evenly distributed, while the stress in the G500-900 and G900-500 scaffolds shows a gradient distribution. The G500-900 scaffold has a small pore size and thick support in the center (red dashed line), which is subjected to more stress during compression. Also, the G900-500 scaffold has a small pore and thickness support on the edge (red dashed line), which increases the load-bearing capacity of the scaffold. As a result, the compression strength of the gradient scaffolds is higher than that of the uniform scaffolds under the same porosity.

**TABLE 3:** Modulus of the elastic modulus of G structural units with different porosities.

Porosity (%)	Elastic modulus (GPa)
20	18.563
30	13.770
40	10.057
50	6.968
60	4.442
70	2.175
80	0.568

**FIGURE 6:** Stress distribution cloud images of the scaffolds under 10% displacement load.

### Phase Structure and Microstructure Analysis

Figure 7 shows the SEM images of the Ni_46.5_Ti_44.5_Nb_9_ scaffold. As seen in Figure 7A, the inside of the scaffold is very dense, no large cracks or inclusions are observed, and only a few voids exist. Figure 7B shows an enlarged image of the red rectangle area in Figure 7A, which clearly shows the melt pool formed by the layer-by-layer build-up with a pool thickness of approximately 30 μm. The microstructure of the scaffold mainly consists of a matrix and round second phase with particle sizes of 10–30 μm. The EDS energy spectra of the matrix and particles (Figure 7C) show that the matrix is mainly NiTi with an Nb content of about 6%, and the particles are Nb particles. This indicates that during the additive manufacturing, part of the Nb is solidly dissolved into the NiTi matrix, forming the solution strengthening. Part of the Nb is retained and uniformly distributed in the matrix, forming second phase strengthening (Liu et al., 2021; Wang et al., 2018). A high magnification image of the Nb particle is shown in Figure 7D, where a fine eutectic structure is formed around the Nb. According to the investigation, the higher cooling rate of the SLM process promotes the diffusion of Nb and produces fine eutectic microstructures, which can improve the strength and ductility of the porous scaffold (Liu et al., 2020).

**FIGURE 7:** XRD pattern and microstructure images: **(A)** microstructure images of the scaffold in the XZ section, **(B)** enlarged image of the red rectangle in **(A**,**C)** and EDS spectrums of points 1 and 2 in **(B**,**D)** eutectic phase and Nb particles.

### Permeability of the Porous Scaffold

Permeability indicates the ability of a fluid to pass through a porous medium and can reflect the ability of the scaffold to transport nutrients and metabolites (Yu et al., 2020). It is an important parameter for biomedical porous scaffolds and is crucial for cell proliferation, differentiation, and the growth of bone tissue (Singh et al., 2009). Figure 8A shows the measured permeability of the scaffolds using the falling head method, and it can be seen that the permeability of the uniform scaffolds gradually increases with the increasing pore size. The G500-900 scaffold with a radial gradient structure exhibits comparable permeability to the G900 scaffold. Figure 8B shows the inlet pressure of the fluid model. The lower inlet pressure indicates that the porous scaffold has less obstruction to the fluid. For uniform scaffolds, the fluid simulation results are the same as for the falling head method, whereas the permeability of the G500-900 and G900-500 scaffolds are comparable to that of the G750 scaffold. It should be noted that the pore size has significantly affected the permeability and the surface area of the scaffolds (Table 1). This is because the surface area of the scaffold decreases with the increasing pore size, which reduces the friction drag of the scaffold during fluid flow, thus increasing the permeability of the scaffold (Ali and Sen, 2018).

**FIGURE 8:** Results of the permeability test and finite element simulation of porous scaffolds: **(A)** permeability test results (the permeability of the G900-500 scaffold is not recorded due to the formation of preparation defects). **(B)** Inlet pressure results are calculated by finite element simulation. **(C)** Fluid pressure distribution cloud diagram. **(D)** Fluid flow velocity distribution diagram. (It should be noted that media of the experiment and simulation are water and human body fluid, respectively).

To investigate the fluid flow inside the porous scaffold, the pressure and flow velocity clouds of the fluid model were the output *via* ANSYS CFD, as shown in Figures 8C,D. In Figure 8C, the section of the uniform scaffold in the axial direction has a stable pressure field, and the pressure gradually decreases, which facilitates the entry of body fluids into the scaffold (Ma et al., 2020). It is worth noting that the G500-900 gradient scaffold has the lowest pressure at the edge in the radial direction, where the scaffold has the largest pore size. This may be the reason why the gradient scaffold has a good comparative permeability with the G750 scaffold. Figure 8D shows the flow distribution of the scaffold. As can be seen, the G500-900 scaffold has the highest flow velocity at the edge, which improves the permeability of the overall scaffold.

## Conclusion

In this study, Ni_46.5_Ti_44.5_Nb_9_ porous scaffolds with different strategies were successfully prepared and simulated by human bone pore size features based on the triply periodic minimal surfaces and selective laser melting technology. The microstructures, mechanical properties, and permeability of the scaffolds were systematically investigated, and the main conclusions are obtained as follows:

1) The Ni_46.5_Ti_44.5_Nb_9_ porous scaffolds have a modulus of elasticity of 0.80–1.05 GPa, a compressive strength of 42.3–65.8 MPa, and an elongation of 15.3–19.1%. For the uniform scaffolds, the pore size strategy has little effect on the mechanical properties of porous scaffolds, and porosity with a continuous gradient distribution can significantly improve the mechanical properties. This is because continuous gradient scaffolds have a low porosity area in the inner or outer regions, and the denser part can bear more stress, thus improving the mechanical properties of the scaffolds.
2) The microstructures of the Ni_46.5_Ti_44.5_Nb_9_ porous scaffolds mainly contain NiTi matrix and Nb particles. The addition of Nb to the NiTi alloy can promote the formation of the eutectic microstructure and precipitation of the rich Nb phase, thus simultaneously increasing the strength and toughness of the alloy.
3) Under the same porosity, increasing the pore size can improve the permeability of porous scaffolds due to the decrease in the specific surface. The local high porosity structure in the continuous gradient scaffolds bears more fluid flow, which can improve the permeability of the overall scaffold.

## Data Availability

The raw data supporting the conclusions of this article will be made available by the authors, without undue reservation.
